# Long-term results after thoracoscopic anterior spondylodesis with or without posterior stabilization of unstable incomplete burst fractures of the thoracolumbar junction: a prospective cohort study

**DOI:** 10.1186/s13018-020-01807-2

**Published:** 2020-09-15

**Authors:** Christof Hoffmann, Ulrich Josef Spiegl, Robert Paetzold, Brian Devitt, Stefan Hauck, Thomas Weiss, Volker Bühren, Oliver Gonschorek

**Affiliations:** 1 Department of Orthopaedic and Trauma Surgery, BG Trauma Center Murnau, Professor Küntscher Str. 8, 82418 Murnau, Germany; 2 Department of Orthopaedics, Trauma Surgery and Reconstructive Surgery, University Hospital Leipzig, Leipzig, Germany; 3 OrthoSport Victoria, Richmond, Victoria Australia

**Keywords:** Thoracolumbar burst fractures, Anterior thoracoscopic spondylodesis, Long-term follow-up

## Abstract

**Background:**

Minimally invasive, thoracoscopic anterior spondylodesis (MIAS) is an established treatment for burst fractures of the thoracolumbar spine. Good restoration of the local sagittal alignment and good functional results have been reported. The aim of this study was to evaluate long-term results of MIAS in patients with incomplete burst fractures and to analyze the influence on global sagittal alignment, clinical outcomes, and adjacent segment degeneration.

**Methods:**

From 2002 to 2003, 18 patients were treated with MIAS for incomplete thoracolumbar burst fractures. Mono-segmental spondylodesis was performed with an iliac crest bone graft and bisegmental spondylodesis with a titanium cage. In this single-center prospective cohort study, 15 patients were available for follow-up (FU) after an average of 12.9 years (12.1–14.4). Seven patients were treated with a combined anterior and posterior instrumentation and eight patients with anterior spondylodesis only. The primary clinical outcome parameter was the Oswestry Disability Index (ODI); secondary parameters were the Short Form 36 (SF36) and the visual analog scale (VAS spine). Full spine radiographs were assessed for bisegmental Cobb angle, alignment parameters, and signs of adjacent segment degeneration (ASD).

**Results:**

ODI evaluation showed a mean impairment of 11.7% with minimal limitations in 13 patients. Neither a significant deterioration over time nor significant differences between both therapy strategies were found in the clinical scores at the latest follow-up. The mean bisegmental increase of regional malalignment of reduction was 8.8° (± 7.3°) with no significant correlation to any clinical outcome scores. The majority of patients had no signs of adjacent segment degeneration. Two patients showed minor radiologic changes. All patients had a balanced sagittal spine profile.

**Conclusions:**

In conclusion, MIAS leads to good clinical results with—in majority—minimal spine-related impairment at the latest follow-up. No significant deterioration at 12-year FU was detectable compared to the 6-year results for the SF36 and VAS spine scores. There was no association between sagittal alignment, clinical outcome scores, and ASD.

**Trial registration:**

The study was retrospectively registered in the German Clinical Trials Register (Nr.00015656).

## Introduction

Incomplete burst fractures of the thoracolumbar junction are common injuries and represent 21% of all burst fractures in this area [1, 2]. Treatment strategies in neurologically asymptomatic patients range from conservative treatment to extensive surgical stabilization [3–7]. No treatment regime has shown superiority; studies comparing operative and non-operative treatment have produced contradictory results [3, 6]. Nonetheless, progressive loss of reduction after posterior only stabilization or non-operative treatment has been reported [5, 6]. It has been suggested that minimally invasive anterior spondylodesis (MIAS) via thoracoscopy, a treatment strategy with a relatively low morbidity, has the potential to improve long-term outcomes [8].

In 2013, Spiegl et al. [9] reported predominantly promising 6-year results and a low complication rate in patients with incomplete thoracolumbar burst fractures. Smits et al. [10] published promising long-term results in 46 patients treated by MIAS. Notably, the overall spinal alignment was not evaluated although this is suggested to represent an important prognostic parameter [11] for long-term success of treatment. Therefore, the aim of this study was to evaluate the long-term outcome of MIAS in patients suffering from incomplete burst fractures of the thoracolumbar junction under consideration of the sagittal alignment. A secondary aim was to analyze the influence of segmental and overall sagittal alignment on clinical outcomes and the potential this may have on adjacent segment disease progression.

Our hypothesis was that MIAS preserves the radiological spinal alignment in the long-term and is associated with good clinical outcomes. A secondary hypothesis was that an increased segmental malalignment would alter the vertebral-pelvic alignment affecting the retroversion of the pelvis which would lead to increased rates of adjacent segment degeneration (ASD).

## Material and methods

This single-center prospective cohort study used the same cohort of patients that was studied previously in a study by Spiegl et al. [9]. Inclusion and exclusion criteria are named in Table 1. One patient was excluded retrospectively from the study as the fracture pattern did not fulfill the inclusion criteria.

**Table 1:** Inclusion and exclusion criteria

Inclusion criteria	Exclusion criteria
➢ Cranial incomplete burst fracture AO type A3.1.1	➢ Prior pathologies at the vertebral spine
➢ McCormack ≥ 6 points	➢ Age < 18 and > 60 years
➢ Thoracolumbar junction: Th10-L2	➢ Contraindication for a thoracoscopic approach
➢ Acute trauma: ventral spondylodesis within 4 weeks after trauma	➢ Posttraumatic neurologic Deficit (ASIA A to D)
➢ High-energy trauma	➢ ASA > 3

All patients suffered from unstable incomplete cranial burst fractures and were treated by MIAS between 2002 and 2003 [9]. The treatment algorithm followed the recommendations of the Spine Section of the German Society of Orthopaedics and Trauma published by Verheyden et al. in 2018 [12]. The protocol, surgical technique, and postoperative rehabilitation have been previously described [9]. Originally, the classification of fracture-type and definition of instability was performed according to Magerl et al. [13] and McCormack et al. [14] by post-traumatic computer tomographic scans. In the current investigation, fractures were re-classified according to the AO spine injury classification system [15]. For anterior spondylodesis, a fixed angle plate (MACS TL, Aesculap, Tuttlingen, Germany) was used on the anterior vertebrae in addition to either a distractable titanium cage (bisegmental, Synex I®, Depuy Synthes, Zuchwil, Switzerland) or autologous tricortical iliac crest bone graft (monosegmental) which was interposed between the vertebral bodies. A typical intraoperative view and operative setting are illustrated in Fig. 1.

**Fig. 1:** Intraoperative view after completion of a minimal invasive monosegmental anterior spondylodesis with a tricortical iliac crest bone graft and MACS plate (**a**) and operative setting (**b**)

In order to release a motion segment, removal of the posterior fixation (Universal Spine System, Depuy Synthes, Zuchwil, Switzerland) was performed in all patients with posterior bisegmental stabilization and anterior monosegmental spondylodesis. This was done at an average of 9.5 months (8–14 months) after the index surgery. In addition to this, one patient who underwent bisegmental anterior-posterior stabilization required implant removal due to irritation of the paravertebral muscles at 3.4 years following the index procedure.

After a minimum of 12 years, the patients were re-evaluated. The primary clinical outcome parameter was the Oswestry Disability Index (ODI) score. The primary radiologic outcome parameter was the bisegmental sagittal increase of malalignment. Secondary clinical outcome parameters were the Short Form 36 (SF-36) domains Physical Component Summary (PCS) and Mental Component Summary (MCS) as well as the VAS spine score (0 = worst pain imaginable; 100 = no pain at all). In addition, patients were asked about their ability to reintegrate back to work, and their symptoms related to the surgical approaches.

The secondary radiological outcome parameters were segmental and overall sagittal alignment parameters as well as radiological evidence of ASD [16] (Table 2). Sagittal alignment was analyzed using the TraumaCAD® Spine 3D-Software (Brainlab Ltd, Israel) in a standardized manner by two investigators on full spine radiographs. In case of fracture of L1, lumbar lordosis was measured from the lower endplate of Th12 to the endplate of S1. Mean intervertebral disc height of the adjacent levels and a reference disc (Fig. 2) were determined according to Spiegl et al. [17]. The disc height was measured postoperatively and at the latest follow-up.

**Table 2:** Radiological signs of adjacent segment degeneration

- 20% or more loss of disc height compared to cranial reference disc	
- Anterolisthesis or retrolisthesis > 3 mm	
- Osteophyte formation > 3 mm

**Fig. 2:** The disc height was measured in the adjacent levels and in a cranial reference level. Disc height was defined as the mean value of the ventral, central, and dorsal disc height

## Statistics

All data were analyzed statistically using the standardized SPSS software 17.0 (SPSS, Inc. Chicago, USA). For statistical analysis of synergies between radiological measurements and clinical outcome parameters a Mann-Whitney *U* test and Kendall’s tau correlation coefficient were used. The level of significance was *p* < 0.05

## Results

Fifteen patients were available for follow-up at a mean of 12.9 years (range 12.1–15.5, individual data are provided in Table 3). Of these, 12 patients presented for clinical assessment, while a further 3 completed their patient-reported outcome measurements. One patient who showed up refused a full spine radiograph. Due to revision of the original CT-scans, one patient was retrospectively excluded from the study as the fracture morphology did not fulfill the inclusion criteria unequivocally. Three patients were lost to follow-up, 2 were uncontactable, and one patient had died in a motor vehicle accident 8 years after the index operation. The clinical findings of the excluded patient and those lost to follow-up at 6 years are displayed in Table 4.

**Table 3:** Patients who were lost to follow-up or excluded from the study retrospectively. Clinical findings at 6-year follow-up

Patient	Age at index operation	Follow-up (year)	Gender	Fracture location	McCormack	AO spine classification	Surgical approach	VB replacement		Follow-up	
									ODI (%)	BiSg Cobb Angle	No follow-up
1	51	13	f	L1	7	A3	Dorso-ventral	Bone graft	14	3	
2	37	12.3	m	L1	7	A3	Dorso-ventral	Bone graft	12	6	
3	42	12.2	f	L1	6	A3	Dorso-ventral	Bone graft	20	5	
4	31	13.9	m	Th12	7	A3	Dorso-ventral	Bone graft	0	~	Only written FU
5	42	15.5	m	L1	7	A3	Dorso-ventral	Cage	10	5	
6	54	12.4	f	L1	8	A3	Dorso-ventral	Cage	0	9	
7	47	13.4	m	L1	7	A3	Dorso-ventral	Cage	0	11	
8	22	12.3	f	L1	7	A3	Ventral only	Bone graft	12	1	
9	23	12.1	f	Th12	6	A3	Ventral only	Bone graft	24	15	
10	52	12.2	m	Th12	7	A3	Ventral only	Bone graft	10	10	
11	31	14.4	f	L1	6	A3	Ventral only	Bone graft	14	~	Refused X-ray FU
12	46	12.5	f	L2	7	A3	Ventral only	Bone graft	4	6	
13	32	12.2	m	L1	6	A3	Ventral only	Bone graft	0	25	
14	43	12.2	f	L1	7	A3	Ventral only	Bone graft	46	~	Only written FU
15	22	12.2	f	L1	6	A3	Ventral only	Bone graft	10	~	Only written FU
16	30	◊	f	L1	7	A3	Dorso-ventral	Bone graft	◊	◊	Wrong address
17	23	◊	f	L1	7	A3	Ventral only	Bone graft	◊	◊	Wrong address
18	36	◊	m	Th12	7	A3	Dorso-ventral	Cage	◊	◊	Died in motor vehicle accident

^◊^Patient lost to follow up

**Table 4:** Clinical findings of the patients who were lost to follow up or excluded retrospectively at 6 year follow up

Treatment strategy	Gender	VAS spine	Reintegration to work	SF36-PCS	SF36-MCS	Donor site morbidity
Anterior-posterior	Female	86	Same job, same intensity	53.09	45.57	Moderate, often
Anterior-posterior	Male	87	Same job, same intensity	24.91	49.38	None
Anterior only	Female	56	Same job, same intensity	35.15	53.57	Slight, infrequent
Anterior-posterior^a^	Female	46	Same job, lower intensity	19.14	62.08	None

^a^Retrospectively excluded patient

### Clinical outcome

ODI evaluation reported a mean spine-related impairment of 11.7% (Table 3). An analysis of the isolated anterior stabilization (anterior_only) and combined anterior and posterior stabilization (combined_AP) subgroups demonstrated comparable long-term results. Thirteen patients had minimal limitations with six patients reporting no spine-related limitations in sports and activities of daily living. One patient reported moderate limitations in the ODI questionnaire (24%) and complained about lasting donor site pain. Overall, three patients complained about lasting donor site-related symptoms. One patient complained about persisting pain in the paravertebral muscles despite posterior implant removal (ODI 10%, PCS 51.9 pts, MCS 54.5 pts). One patient was severely limited (ODI 46%) and had to change work due to back pain (VAS spine 35.2) and donor site symptoms; this patient reported severe limitations with an ODI of 46%. Notably, this individual had suffered a polytrauma (Injury Severity Score of 19) at the index presentation, which included extensive abdominal injuries (splenic rupture, small-intestine rupture) and fracture of the upper extremities (fracture of distal radius AO type 23C3.3). The postoperative symptoms were not exclusive to the patient’s back issues but also related to abdominal discomfort and upper extremity symptoms.

SF 36 score evaluation showed a mean overall PCS score of 42.4 (± 12.1), and a mean MCS of 51.4 (± 8.1) (Fig. 3). No statistically significant differences could be found between the PCS and MCS scores at 6-year follow and at long-term follow-up (mean 12.9 years). Also, there was no significant difference between the long-term result of the current study and the results of a control group of the same age (50–59 years, MCS 49.1 (48.4–49.8); PCS 50.4 (49.9–51.0) [18]). Figure 4 illustrates the VAS spine score results at 6 and 12 years follow-up. Altogether, fifteen patients were able to maintain work without any limitations.

**Fig. 3:** Overall PCS and MCS results at 6- and 12-year follow-up. The numbers in the figure represent the corresponding patients the table

**Fig. 4:** The course of the VAS spine score of the 15 patients who were available for follow-up

### Radiological outcome

Preoperative regional kyphosis, operative reduction, and the chronological sequence of the bisegmental Cobb angle are shown in Fig. 5. Global and regional alignment parameters are shown in Table 5. Regional and global parameters showed balanced spine alignment and no significant correlation to the bisegmental sagittal increase of regional malalignment. No significant correlation was found between alignment parameters and clinical outcome scores. With the exception of one lymphoma-induced pathologic fracture (TH8), no subsequent vertebral fracture was identified. Figure 6 exemplifies long-term radiological findings after anterior monosegmental spondylodesis with a tricortical iliac crest bone graft and MACS-plate.

**Fig. 5:** Time course of regional sagittal alignment parameters

**Table 5:** Sums up the radiological findings according to the treatment strategy

**Fig. 6:** Full spine radiograph showing long-term radiological follow-up after monosegmental anterior spondylodesis with a tricortical iliac crest bone graft and MACS plate. Plate osteosynthesis of the iliac crest was performed to restore the shape of the iliac crest

No significant difference was found in relation to disc height or loss of disc height in the adjacent levels between the different operative strategies. Two patients displayed the formation of new osteophytes (> 3 mm in size) in the adjacent segments, but there was no association with anterior or posterior spondylolisthesis. No relevant loss of disc height (> 20% compared to a cranial reference disc) was found in the cohort. Furthermore, no significant correlation was found between the loss of disc height and increase of regional malalignment.

## Discussion

The most important finding of this study was that patients who underwent MIAS for incomplete burst fractures of the thoracolumbar spine had mainly good to excellent long-term clinical outcomes. Specifically, a comparison of the medium (6 year) and long-term (12 year) clinical outcomes revealed no deterioration. Overall, spine-related impairment remained low in the majority of patients with no significant difference between the surgical treatment of anterior only and combined anterior and posterior stabilization. Furthermore, radiological findings demonstrated that the segmental and overall alignment parameters were unchanged over time. All patients presented with perpendicular sagittal profiles and no radiological signs of decompensation. These findings indicate that MIAS is an effective and reliable technique with lasting long-term results for the treatment of incomplete burst fractures of the thoracolumbar spine.

### Clinical outcome

In this investigation, ODI evaluation reported a mean impairment of 11.7%, which equates to minimal disability at the latest follow-up of 12 or more years. Unfortunately, these results cannot be compared over time as ODI was not evaluated at the time of patient inclusion and at the 6-year follow-up. However, it is encouraging that these scores mimic the values reported by Scholz et al. [7] in a short-term follow-up (2 years) of patients treated with a combined anterior and posterior stabilization using the MIAS technique (ODI score of 13.3%). These positive results were reinforced by an analysis of the SF 36 domains in our study demonstrating no differences between the 6- and 12-year follow-up as well as in comparison to a healthy control group of the same age.

Notwithstanding, non-operative treatment is a generally accepted treatment alternative for incomplete burst fractures of the thoracolumbar junction without neurologic deficits [3]. Thereby, Wood et al. [3] presented favorable long-term clinical results for non-operative treatment of thoracolumbar A3/A4 fractures. They presented a median ODI score of 4% after a follow-up of 18.6 years for those treated non-operatively whereas the cohort treated operatively had a median ODI score of 40%. However, despite the better clinical outcome following non-operative treatment, a relevant bisegmental sagittal loss of reduction was observed in this collective with an average Cobb angle of 19° (10–29°). This might lead to a decompensated sagittal alignment in the future with associated symptoms. Interestingly, Wood et al. [3] reported on far higher rates of ASD of 70% in the non-operative group and 64% in the operative-treated group compared to 15% in our patient population.

Two further studies reported on long-term outcome after non-operative treatment of thoracolumbar burst fractures. Weinstein et al. [19] re-evaluated 42 patients with thoracolumbar burst fractures at a mean follow-up of 20 years. They found an average Oswestry Low Back Pain Score of 3.5 in a heterogeneous cohort of thoracolumbar and lumbar fractures. Taking into account that we used a VAS spine score with an inverted scale, these findings are slightly worse than the results of our cohort. Further, Moller et al. [20] followed 27 patients with a 23–41 year follow-up. Twenty-one patients (78%) showed a mean ODI score of 8% demonstrating a slightly better clinical outcome compared to our cohort. However, Moller et al. reported on a heterogeneous collective with a wide range of fracture location and fracture morphology with a follow-up rate of only 51%. Although the average bisegmental kyphosis was reported to be > 20°, there was no correlation between alignment and clinical outcome. In summary, a clearly superior regional long-term alignment is visible in our patient collective treated surgically using MIAS compared to a non-operative therapy. However, we could not proof a clinical benefit of our surgical strategy. This might be caused by our inclusion criteria of unstable fractures with a load sharing classification of 6 and higher [14]. Further matched-paired or randomized control trials need to evaluate this important question in more detail.

Additionally, the proportion of patients complaining about approach-related symptoms after iliac crest harvesting remained high which might explain the slightly inferior clinical results. Three patients complained about pain or hyposensitivity at 12 year follow-up. At 6-year follow-up, 71% of all patients were suffering from donor site pain [21]. These findings are consistent with the findings of Wippermann et al. [22] who reported an overall complication rate of 19.6% after iliac crest harvesting. Based on these results, the authors do not implant iliac crest grafts any longer. We changed our therapy regime to trabecular metal cages for monosegmental and distractable titanium cages for bisegmental vertebral body replacement. At 12-year follow-up, the morbidity of the anterior thoracoscopic approach was still negligible with only one patient complaining about mild regional hyposensitivity.

### Radiologic outcome

In our cohort, radiographic examination revealed a moderate bisegmental increase of regional malalignment of 9° at the latest follow-up. Progression of regional malalignment after complete bony healing is surprising at first sight. We believe this can be explained by a continuous loss of vertebral disc height in the adjacent motion segments on the one hand and by an ongoing remodeling process of the bone graft in patients treated with monosegmental spondylodesis on the other hand. Low to moderate cage subsidence might explain this situation in patients treated bisegmentally. Interestingly, there was a higher increase of regional malalignment in the anterior_only group compared to the combined_AP stabilized group. This might be caused by the improved initial reduction after combined_AP treatment. However, the differences were not found to be significant, although this may be due to the small sample size.

Recently, Smits et al. [10] reported promising results in 46 patients with thoracolumbar fractures treated by MIAS at a median follow-up of 49 months. Thereby, the overall bisegmental loss of reduction in this cohort was comparable to our results with a mean of 6.8°. However, Smits et al. did not investigate the effects of the MIAS technique on spinal alignment and included a more heterogeneous group of patients with a diverse variety of fracture types, neurological status, fracture locations, and time to follow-up.

In contrast, Scholz et al. [7] found a mean loss of reduction of only 1.9° in the combined_AP treated subgroup. This lower loss of reduction might be caused by the far shorter follow-up of only 2 years. Similarly, in the previous investigation of our cohort, Spiegl et al. [9] reported a loss of reduction of 4.0° at 18 months follow-up but reported a relevant progression in the further course after removal of the posterior implants. Korovessis et al. [5] reported a mean bisegmental loss of reduction of 2° over 46 months in a combined_AP stabilized cohort and a mean loss of 5° over 48 months in a posterior only stabilized subgroup with mid-lumbar A3 fractures. Hereby, the reduced loss of reduction can be explained by the fracture location at the lordotic mid-lumbar spine.

Additionally, a higher reduction loss can be caused by the implantation of autografts in the majority of our patients. Lack of intrinsic stability of iliac crest bone grafts and loss of height due to late onset bony healing are possible reasons for a worsened radiologic outcome [21]. In combination with frequent donor site symptoms, this led to a replacement of autografts by cages in our department.

### Adjacent segment degeneration

ASD is an acknowledged problem after segmental spinal fusion in treatment of degenerative disc disease [23, 24]; increased movement and mechanical loading on the adjacent discs are potentially causative factors. After definition of radiologic signs of ASD, Tsuji et al. [16] reported 21 cases of ASD in a cohort of 71 patients who underwent PLIF-operation after 5 years. Although the underlying conditions are not directly transferable, ASD might be a long-term problem after trauma-related spinal fusions, too. As previously reported, Wood et al. [3] reported on rates of ASD of 64% in the intervention group and 70% in the non-operative group in trauma patients. However, Wood et al. [3] did not define limit values for radiological signs of ASD in detail. In our study, we found new onset of osteophytes in the adjacent segments in two out of 12 patients. Other signs of degeneration like disc space narrowing or listhesis were not observable. One possible reason for this relatively low rate of ASD is the younger average age of our patients collective at final follow-up (52 years vs 62 years Wood et al.). However, the most likely parameter for ASD progression is the high regional malalignment considering the high kyphotic Cobb angle of 19° in the latest follow-up.

Overall, no statistically significant correlations between alignment parameters and clinical outcome scores could be found. These results are in accordance to other studies which state that patients do not necessarily present with a clinical deterioration in cases with mild to moderate kyphotic malalignment [5, 19]. However, Gertzbein et al. [25] found significantly higher rates of back pain in patients with kyphotic malalignment of more than 30°. In our cohort, the mean loss of reduction was 9° which might be too small to affect compensation mechanisms, and the maximum kyphosis of 22° was also lower than the critical amount of 30° [25]. All patients showed balanced sagittal alignment parameters with a perpendicular spine profile. Overall, the interpretation of effects remains difficult due to a wide range of data and variations between individuals [26].

### Limitations

The major limitation of this study is the low number of included patients. Thus, the study might be under-powered to detect differences between the anterior only and combined anterior and posterior therapy strategy. However, the main purpose of this study was to evaluate long-term clinical und radiological results of MIAS in a highly specific patient group (affected vertebral bodies of the thoracolumbar junction only, acute A3 fracture, no osteoporosis). The authors were particularly interested in evaluating approach-related symptoms and analyzing the long-term effect for ASD progression and sagittal alignment.

Additionally no randomization has been performed leading to an inhomogeneous distribution of fracture types and grades of instability between the two subgroups in the index study. Hereby, it would be interesting to compare the anterior only strategy with a combined anterior and posterior treatment in a bigger patient population.

Furthermore, clinical investigation and full spine radiographs were not available in all cases at the latest follow-up. Besides, sagittal alignment and the results of the ODI evaluation cannot be put in a chronological correlation as both had not been used in the preceding investigation. However, both the ODI score and full spine radiographs were not commonly evaluated in 2002. Besides, two different operative strategies (anterior_only vs combined_AP) were used and, in the meantime, the operation technique for MIAS using iliac crest bone crafts had been widely replaced with titanium cage implementation.

However, the strengths of this study are the prospective data acquisition and the high comparability of the analyzed fractures as only A3 fractures of the thoracolumbar junction were included. Loss of follow-up was excellent with less than 20% over 12 years.

## Conclusion

In conclusion, MIAS leads to good clinical results with—in majority—minimal spine-related impairment at the latest follow-up. No significant deterioration at 12-year FU was detectable compared to the 6-year results for the SF36 and VAS spine scores. There was no association between sagittal alignment, clinical outcome scores, and ASD.

## Data Availability

The datasets used and analyzed during the current study are available from the corresponding author on reasonable request.

## Abbreviations

~: No radiologic follow-up available
◊: Patient lost to follow-up
Anterior_only: Isolated anterior stabilization
Age: Age at index operation
ASD: Adjacent segment degeneration
AO: Arbeitsgemeinschaft für Osteosynthesefragen
AP: Anterior-posterior
BiSg: Bisegmental
Combined_AP: Combined anterior-posterior stabilization
f: Female
L: Lumbar vertebra
Loc: Location
m: Male
MCS/MSC: Mental component summary
MIAS: Minimally invasive anterior spondylodesis
MonoSg: Monosegmental
ODI: Oswestry Disability Index
PCS/PSC: Physical Component Summary
pts: Points
S: Sacral vertebra
SF36: Short Form 36
SVA: Sagittal vertical axis
TH: Thoracic vertebra
VAS: Visual analog scale
VB: Vertebral body
